The article "A histopathological analysis of the epidemiology of coronary atherosclerosis: an autopsy study" was retracted in 2016. Reasons: plagiarized text; compromised peer review; false authorship.

# A histopathological analysis of the epidemiology of coronary atherosclerosis: an autopsy study

**DOI:** 10.1186/s13000-015-0324-y

**Published:** 2015-07-03

**Authors:** Negin Abedinzadeh, Behnam Pedram, Yasan Sadeghian, Seyed Mohamad Hossein Tabatabaei Nodushan, Maryam Gilasgar, Mahsa Darvish, Aram Mokarizadeh

**Affiliations:** Graduate, Faculty of Medicine, Tehran University of Medical Sciences, Tehran, Iran; Department of Pathobiology, Susangerd Branch Islamic Azad University, Susangerd, Iran; Graduate, Faculty of Medicine, Shahid Beheshti University of Medical Sciences and Health Services, Tehran, Iran; Cellular & Molecular Research Center, and Department of Immunology, Kurdistan University of Medical Sciences, Sanandaj, Iran

**Keywords:** Atherosclerosis, Coronary artery, Autopsy, Inflammation, Plaque

## Abstract

**Background:**

Atherosclerosis accounts for a large proportion of cardiovascular system associated morbidity and mortality. We studied the possible association between the histopathological changes of the coronary atherosclerotic lesions and the risk of sudden cardiac death (SCD) using autopsy cases.

**Methods:**

We performed an autopsy analysis (n = 13, 4 women, 9 men mean age 67.5 years; age range 56–93 years) of SCD which occurred in patients aged over 50 years during March 2010 to December 2013. The following variables were considered: sex, age, medical history, autopsy findings to macroscopic and histological evaluation of the heart. The autopsies were performed according to standard techniques. In all subjects, the heart was dissected following standard autopsy protocol and a 5 cm section of the right coronary artery (RCA) in the atrio-ventricular groove from its origin, a 5 cm segment of the left anterior descending artery (LADA) distal to the origin of the circumflex artery, but including the region of origin of the circumflex branch and left coronary artery (LCA) from its origin till the circumflex branch were excised, dissected out, fixed in 10 % formalin, marked for identification and sent for histopathological analysis.

**Results:**

Atherosclerotic plaques were identified in 6.5 % of specimens, 69.34 % of males and 30.66 % of female. Such plaques were typically concentric and more represented with necrosis, calcification, cholesterol crystals, and giant cells, as well as had a higher inflammatory cell count. Furthermore, intima and media thickness of coronary arteries were significantly higher in studied specimens with visualize the connective tissue layers of the adventitia and the fatty acid containing adipose cells in the periadventitial tissue. Furthermore, the degree of microscopic lesion of atherosclerosis increased proportionally with the increase in the intensity of lipid deposition and with the percentage of collagen in the atherosclerotic plaques.

The article "A histopathological analysis of the epidemiology of coronary atherosclerosis: an autopsy study" was retracted in 2016. Reasons: plagiarized text; compromised peer review; false authorship.

**Conclusion:**

In this study, age estimate to be a risk factor for coronary atherosclerosis in individuals more than 50 years old and may be used to predict SCD. Altogether, an enhanced understanding of the pathobiologic processes responsible for atherosclerotic changes might allow for early identification of a high-risk coronary plaque and thereby provide a rationale for innovative diagnostic and/or therapeutic strategies for the management of coronary patients and prevention of acute coronary syndromes.

## Background

Coronary artery disease (CAD**)** is a leading cause of death of women and men worldwide. An estimated 17.5 million people died from this cause in 2005, representing 30 % of all deaths in the world; of these, 7.6 million were caused by coronary heart disease [1]. Aging is associated with structural and functional changes of the vessel wall, which result in decreased vascular distensibility and elevated arterial stiffness [1, 2]. As a consequence of arterial stiffness, systolic blood pressure increases, causing a rise in left ventricular workload and subsequent hypertrophy, and diastolic blood pressure decreases, leading to an impaired coronary perfusion [2, 3]. Chronic systemic inflammation has been implicated in atherogenesis, and may play a role in destabilizing vulnerable coronary plaques, thereby precipitating acute thrombosis and clinical coronary vessel events [4].

Atherosclerosis is a pathologically diverse disease with heterogeneous mechanisms of progression. Irreversible atherosclerotic plaques begin with smooth muscle cell-rich lipid pool lesions referred to as pathologic intimal thickening and it is a lipid-driven, chronic inflammatory disease of the vessel wall in which both innate and adaptive immune responses play a role. Moreover, atherosclerosis is a complex process involving inflammation and cellular proliferation in the arterial wall that is mediated by a variety of growth factors, cytokines, thrombotic factors, and vasoactive molecules [7]. Mature lesions exhibit calcification [5], which is mediated by cells similar to osteoblasts [6, 7]. Infectious agents may be involved in the initiation and/or progression of atherosclerotic lesions [8]. Roles have been suggested for a host of other factors in the etiology of atherosclerosis and of clinical events [9], including hemostatic factors [10, 11], factors related to lipoprotein metabolism, insulin resistance [12], homocysteine [4], immune factors [13], inflammation markers [14], specific fatty acids [15, 16], indicators of oxidative stress, and circulating markers of endothelial function such as cellular adhesion molecules and thrombomodulin [17].

The article "A histopathological analysis of the epidemiology of coronary atherosclerosis: an autopsy study" was retracted in 2016. Reasons: plagiarized text; compromised peer review; false authorship.

Coronary calcium is a specific marker of atherosclerosis [18] that has been included in the Coronary Artery Risk Development in Young Adults Study [19] and in subgroups in the Atherosclerosis Risk in Communities Study and the Cardiovascular Health Study [20]. Coronary artery calcification (CAC) is a linear estimate of the total burden of coronary atherosclerosis that highly correlates with autopsy and intravascular ultrasound assessment [21]. In fact, CAC provides a better estimate of burden of disease than luminal stenosis as determined by angiography [22], since less-obstructive plaques actually give rise to more occlusions than more-obstructive plaques because of their greater number. In fact, 70 % of patients with acute MI have stenosis of less than 50 % in their culprit artery on angiography [23]. Therefore, stress testing (treadmill, nuclear medicine, or echo), which typically diagnoses the physiological effects of high-grade stenosis, will fail to identify a significant number of persons at risk for a hard event [24]. CAC detection by computed tomography directly detects only hard or calcified plaque, but the calcification found essentially serves as a surrogate marker for soft or non-calcified plaque as well, since in the vast majority of patients both types of plaques coexist proportionally [25]. It should be noted that no current imaging test is able to identify plaque that is prone to rupture, and that the presence of calcification in a coronary artery does not necessarily indicate a stenosis at that site; the value of CAC assessment is, rather, in its ability to reflect the overall burden of coronary atherosclerosis.

The objective of the study was to determine the possible association between the histopathological changes of the coronary atherosclerotic lesions and the risk of sudden cardiac death (SCD) and acute myocardial infarction (AMI) using autopsy cases.

## Methods

This study was conducted from March 2010 to December 2013 in the General Mortuary based at the Tehran forensic medicine center with various causes of death (sudden cardiac death and myocardial infarction).

### Study objects and specimen preparation

This study was approved by the local ethics committee. The hearts of 13 patients (4 women, 9 men mean age 67.5 years; age range 56–93 years) were collected at autopsy within 8 h after death. Inclusion criteria were age over 50 years and an autopsy had to be intended. All cause of death were sudden cardiac death and acute myocardial infarction (n = 13). A signed letter of consent was taken from the relatives of the dead bodies. Human hearts were obtained from a pathologic study of sudden cardiac death due to atherosclerosis and coronary artery thrombosis. After explanation from the corpse, the hearts were washed in water without further fixation or staining.

The article "A histopathological analysis of the epidemiology of coronary atherosclerosis: an autopsy study" was retracted in 2016. Reasons: plagiarized text; compromised peer review; false authorship.

### Preparation of the coronary arteries

The heart was dissected following standard autopsy protocol at autopsy. The coronary arteries were cannulated, washed with 0.1 mol/L PBS (pH 7.4), and perfused with 1 L of freshly prepared 4 % (wt/vol) paraformaldehyde in 0.1 mol/L sodium phosphate (pH 7.4) at 100 mmHg. Next, the heart was immersed in 4 % paraformaldehyde for at least 24 h at 4°C. A 5 cm section of the right coronary artery (RCA) in the atrio-ventricular groove from its origin, a 5 cm segment of the left anterior descending artery (LADA) distal to the origin of the circumflex artery, but including the region of origin of the circumflex branch and left coronary artery (LCA) from its origin till the circumflex branch were excised and dissected out. All the sections of coronary arteries from each case were fixed in 10 % formalin, marked for identification and sent for histopathological analysis. Paraffin sections were made and the sections stained using Hematoxylin and Eosin (H & E) dyes.

### Histopathological examination

In all subjects, the heart was fixed with 10 % formalin. All specimens of coronary arteries were taken from each heart for histopathological examination. Twenty-six blocks from the right and left coronary artery were cut into 5-μm-thick serial sections and each section was stained with hematoxylin and eosin stains. When necessary, samples were partially decalcified by acid extraction before sectioning. The atherosclerotic lesion type of each section was carefully classified by 2 investigators simultaneously using a double-headed light microscope.

### Grading atherosclerosis by pathologists

Two pathologists independently estimated the percentage of the tunica intimal and medial surfaces area involved with fatty streaks and raised lesions in the coronary arteries. The consensus lesion grade was the average of the grades of 2 pathologists and raised lesions mostly included an area of hemorrhage, thrombosis, ulceration, or calcification.

## Results

Histopathologically, moderate to severe atheromatous lesions were observed in the coronary arteries. The subendothelial space was dilated by an extracellular network containing large amounts of fibrin/collagen composite materials in sections stained with H&E.

In some cases, a numerous number of macrophages and occasionally lymphoplasmacyte-rich infiltrates were detected in the subendothelial space with lipid deposition (Fig. 1a and Fig. 2d). The intimal and medial smooth muscle cells usually had swollen nuclei and abundant cytoplasm. In most cases, severe atheromatous lesions containing abundant chronic inflammatory cells infiltration (Lymphocytes were the dominant inflammatory cells) and calcium deposits were frequently observed in the tunica media and adventitia of coronary arteries (Fig. 3d). These histologic changes were consistent with atherosclerotic deposits, early aneurysm formation, and chronic and acute hemorrhage (Fig. 1b and 1d).

The article "A histopathological analysis of the epidemiology of coronary atherosclerosis: an autopsy study" was retracted in 2016. Reasons: plagiarized text; compromised peer review; false authorship.

**Fig. 1:** Micrographs showing the coronary tree from patients who died of acute myocardial infarction (AMI) . Panel (**a**) demonstrates the fatty deposits in adventitia and inflammatory cells surrounding the media of this arteriole are seen (H&E, 200 Ҳ). Panel (**b**) shows the deposition of lipids and infiltration of lipid-laden foamy cells in the tunica intima and tunica media together with severe narrowing by atherosclerotic plaque, with several hemorrhagic necrotic cores (H&E, 400 Ҳ). Panel (**c**) indicates histologic finding with fibrous tissue, and necrotic core (H&E, 400 Ҳ). Panel (**d**) shows microscopic section of the coronary artery shows thickening of the vascular wall by atherosclerotic deposits and hemorrhage. (H&E, 200 Ҳ)

**Fig. 2:** Micrographs showing the three major epicardial coronary arteries from patients from the who died of a sudden cardiac ischemic death. Panel (**a**) demonstrates severe atheromatous lesions, calcium deposits of luminal atherosclerotic plaques with hemorrhage, hyaline material in the tunica media (H&E, 200 Ҳ). Panel (**b**); Photomicrograph of a coronary plaque (H&E stain) showing intraplaque hemorrhage with the necrotic core with a form of calcification that result in irregular nodules of calcium (H&E, 200 Ҳ). Panel (**c**) indicates a prevalently fibrous plaque characterized by a necrotic core associated with a thick fibrous and this photograph of coronary plaques demonstrates multiple necrotic cores (H&E, 400 Ҳ). Panel (**d**) shows occasionally lymphoplasmacyte-rich infiltrates and fibroproliferative tissue together with areas of free cholesterol crystals (H&E, 400 Ҳ)

**Fig. 3:** Histopathological localization of atherosclerotic lesions of the human coronary artery. Panel (**a**) shows the bright luminal fibrous layers in the atherosclerotic plaque with the resolution obtained together with the minimal obstruction to the coronary lumen caused by atherosclerotic plaque (H&E, 200 Ҳ). . Panel (**b**) Magnification × 200, H&E stain. An un-normal coronary wall. Note thickened media, which contained cholesterol crystals within the tunica media together with lesions with fibromuscular fibrous. Panel (**c**): Photomicrograph of thick part of atheroma and shows extracellular lipid forms a confluent core in the musculoelastic layer of eccentric adaptive thickening that is always present in this location and the lipid core also contains cholesterol crystals and dark staining aggregates of microcrystalline calcium (H&E, 400 Ҳ). Panel (**d**) demonstrates severe atheromatous lesions containing abundant lymphocytes cells infiltration and the deposition of lipids and infiltration of lipid-laden foamy cells in the tunica intima and tunica media (H&E, 400 Ҳ)

Numerous macrophages with foamy cytoplasm infiltrated the tunica intima and media (Fig. 2a). In severe lesions, the tunica media contained enlarged macrophages with foamy cytoplasm, hyaline material, fibrofatty plaque. and mineralized material (Fig. 2a). The lesions were characterized by the deposition of lipids and infiltration of lipid-laden foamy cells in the tunica intima and tunica media, sometimes forming fibrofatty plaques (Fig. 1b), containing abundant cholesterol clefts (Fig. 2d and 3b) and mineralized material. The lesions started in the tunica intima and extended to the tunica media and tunica adventitia. In some cases, lesions were characterized by dense intimal fibrosis with necrotic debris and (Fig. 1c and Fig. 2c) foam cells typical of atherosclerosis. Restenotic lesions were characterized by an increased proportion of loose fibroproliferative tissue, as well as all types of lesion pathology were observed in proximal, mid, distal and branch segments in these 13 cases. However, proximal lesions were more commonly atheromatous plaques (Fig. 3a and 3b) as compared with distal narrowing’s.

The article "A histopathological analysis of the epidemiology of coronary atherosclerosis: an autopsy study" was retracted in 2016. Reasons: plagiarized text; compromised peer review; false authorship.

Moreover, the combination of densely layered collagen and degenerating tissue was significantly more common in specimens from pathologic lesions, whereas loosely arranged proliferative tissue was significantly more common in tissue from atherosclerotic lesions (Fig. 3c). Furthermore, the study has revealed that ruptured plaques of human autopsied affected were characterized by the presence of a more severe inflammatory infiltrate (Fig. 1a), constituted by monocytes, macrophages, and lymphocyte cells. Areas of necrosis and the existence of giant cells were also more frequent in segments with luminal atherosclerotic plaques. Inflammatory cells were more abundant within segments with luminal atherosclerotic plaques (Fig. 3d). Calcium deposits were more commonly seen in segments containing luminal atherosclerotic plaques (Fig. 2a). Whereas the presence of calcium deposits had an excellent specificity of luminal atherosclerotic plaques, the majority of atherosclerotic plaques (Fig. 3a and 3b) were not calcified, and hence, sensitivity was much lower. Although we had not stained the internal elastic lamina because of extreme superficiality of the calcified areas, we supposed that most of them were intimal in location. In the present study, calcium in the coronary plaque is often fragmented and may be located deep in the plaque or close to the surface (Fig. 3c). However the frequency of calcified nodules (with surface thrombus), a form of calcification that results in irregular nodules of calcium (Fig. 2b), is higher in coronary disease.

The article "A histopathological analysis of the epidemiology of coronary atherosclerosis: an autopsy study" was retracted in 2016. Reasons: plagiarized text; compromised peer review; false authorship.

Finally, the most important findings were the presence of pseudocalcium–calcium (pCa–Ca) deposits and arterial wall degeneration. Proliferative lesions have been found in the coronary arteries of thirteen specimens of human autopsy. In the present study, 69.34 % of male showed atherosclerosis and 30.66 % of female showed atherosclerosis.

## Discussion

Atherosclerosis is a disease of large- and medium-sized muscular arteries, characterized by inflammation of smooth muscle cells and formation of atherosclerotic plaques composed of necrotic cores; calcium deposits; and an accumulation of modified lipids, endothelial cells, leukocytes, and foam cells [26–31]. Many components of the vascular, metabolic, and immune systems are involved in this process [27, 30, 32–36]. Buildup of material and infiltrates leads to vascular remodeling, acute and chronic luminal obstruction, abnormalities of blood flow, and diminished oxygen supply to target organs [27, 28, 34]. In human beings, atherosclerosis is the most common pathologic process leading to cardiovascular disease [34–36].

The autopsy study provides a means of understanding the basic process which sets a stage for clinically significant atherosclerotic cardiovascular disease. There is no valid method of sampling of living population. It was, therefore, considered that death suspected due to cardiovascular pathology, probably provide the best sample of the living population for studying atherosclerosis.

In this study, the histological examination of the serially sectioned coronary arteries from 13 men and women who died suddenly and unexpectedly revealed the frequent presence of early atherosclerotic lesions in 13 cases. The lesions are marked by infiltration in the intima and media of coronary artery, monocytes/foam cells, rich-lymphocytes and deposits of mineral material, mainly composed of cellular matrix network, as well as fragmentation of the elastic fiber system.

Age is a powerful risk factor for coronary heart disease. The development of atherosclerosis increases markedly with age up to an age of about 65, regardless of sex and ethnic background [37, 38]. The autopsy findings of coronary arthrosclerosis in different reports are variable in relation of age and sex. In an autopsy study by Thomas et al. [39] among 124 men (age range, 50 to 69 years) who died of non - cardiac causes, 10.3 % had one-vessel, 2.8 % had two-vessel, and 1.4 % had three-gmale in age group between 52 and 83 years. This prevalence of coronary atherosclerosis is higher but supported by other investigators. The coronary atherosclerosis is also increasing with rapid pace in older age group also.

The article "A histopathological analysis of the epidemiology of coronary atherosclerosis: an autopsy study" was retracted in 2016. Reasons: plagiarized text; compromised peer review; false authorship.

Autopsies performed on casualties of the Korean War revealed coronary artery involvement in 77.3 % of the hearts studied, and data after the Vietnam War noted the presence of atherosclerosis in 45 % of casualties with severe disease in 5 %. One hundred eleven victims of non-cardiac trauma underwent pathologic examination of their coronary arteries to estimate the presence and severity of coronary atherosclerosis. Sudden coronary death (SCD) in older individuals is generally associated with extensive coronary atherosclerosis, although it may be the first manifestation of ischemic heart disease. In younger age-groups, SCD may occur in the presence of less severe disease [40].

Low-density lipoprotein remains the most important risk factor for development of atherosclerosis in humans and has been also associated with atherosclerosis in animals [27, 29, 34, 35]. However, immune and inflammatory mechanisms of atherosclerosis have gained tremendous interest in the past 20 years [28–30, 35, 36]. New data suggest an important role for chemokine’s and chemokine receptors in atherosclerosis and highlight a network of cytokines that modulate the immune response and inflammation of the arterial wall [30, 31]. Because it has been shown in humans that all phases of atherosclerosis are regulated by inflammatory mechanisms, the possible impact of chronic inflammation in the development of atherosclerosis in animals and the importance of preventive diagnosis should be considered [30, 31].

In our study, an increased number of inflammatory cells, the presence of giant cells and areas of necrosis and calcification were more frequent in segments containing atherosclerotic plaques, consistent with findings from studies on atherosclerosis of coronary arteries [41–43]. Moreover, lymphocytes were more abundant in sections containing atherosclerotic plaques. However, contrary to what has been reported from the analysis of arterial plaques [43], in our study, lymphocytes were the predominant inflammatory cells in the majority of atherosclerotic plaques. The findings of a study by van der Wal et al. [44] also suggested a predominance of lymphocytes in venous compared with arterial plaques. Although the reasons for a predominance of lymphocytes in vessel atherosclerotic lesions need further investigation, it has been suggested that dendritic cells and lymphocytes co-accumulate in atherosclerotic vein grafts, suggesting an immune-mediated antigen presentation to lymphocytes [45]. It might be the case that in human venous plaques, lymphocytes are dominant inflammatory cells that render the venous plaques more vulnerable to rupture or disruption because of interferon- production, which reduces the fibrous cap thickness [41, 42].

The article "A histopathological analysis of the epidemiology of coronary atherosclerosis: an autopsy study" was retracted in 2016. Reasons: plagiarized text; compromised peer review; false authorship.

In the present study, it was observed that nine cases (69.34 %) were males and 4 (30.66 %) were females, which are concordant with other researchers findings that showed 74.8 % males and 24.2 % females, and another study found 66.5 % males and 33.5 % females [46, 47]. In the present study, 69.34 % of male showed atherosclerosis & 30.66 % of female showed atherosclerosis which are concordant with the study of Thej et al., showed 62 % were males & 50 % were females in Indian population [48]. Study reported by Yazdi SAT et al., showed 73 % males and 61 % females had atherosclerosis in a population of Iran. This difference is again explained by the demographic, geographic, racial, lifestyle & dietary variation in population [49] Singh H et al., have reported the incidence of atherosclerosis in the coronaries to be 68 % in males and 27 % in females [50].

Coronary artery calcium (CAC) has been demonstrated to be associated with the risk of coronary heart disease. Our study showed that the information provided here can be used to examine whether a patient has a high CAC score relative to others with the same age, gender, and race/ethnicity who do not have clinical cardiovascular disease or treated diabetes. Rumberger et al. have made additional recommendations for specific cut points for mild, moderate, and severe coronary artery calcium that have been used frequently in clinical practice [51]. The ACC/ In contrast, a “high” calcium score indicates greater likelihood of disease and may be consistent with moderate to high risk of a cardiovascular event during that time period. However, some post-mortem pathologic analyses of coronary arteries reported that calcium was a frequent feature of plaque rupture [52, 53]. Other reports have been shown that ruptured plaques were less likely to be calcified in acute coronary syndrome patients [54, 55]. Thus, coronary calcium is not a marker for neither unstable nor stable plaques.

If calcium does have a different impact on risk depending on race, then the observed CAC should be evaluated relative to subjects of the same age, gender, and race/ethnicity, as presented here. It is premature to use percentiles from either this study or others to make medical decisions. In other words, at this time, the information presented here cannot necessarily be used to conclude that a patient is “high risk” but can indicate whether they have a high calcium score relative to others with the same age, gender, and race/ethnicity [56–59].

The article "A histopathological analysis of the epidemiology of coronary atherosclerosis: an autopsy study" was retracted in 2016. Reasons: plagiarized text; compromised peer review; false authorship.

Atherosclerosis and coronary artery disease are huge health concerns in Iran. They constitute the largest single cause of death and exact a financial burden of billions of dollars annually. It is well known that lifestyle modification and drug therapy in selected individuals can reduce the risk of hard cardiac events, but current Framingham risk assessment is suboptimal.

## Conclusions

Our study suggested that although calcification is found more frequently in advanced lesions, it may also occur in small amounts in earlier lesions, which appear in the second and third decades of life. Histopathological investigation has shown that plaques with microscopic evidence of mineralization are larger and associated with larger coronary arteries than plaques or arteries without calcification. The relation of arterial calcification to the probability of plaque rupture is unknown. Although the amount of coronary calcium correlates with the amount of atherosclerosis in different individuals and to a lesser extent in segments of the coronary tree in the same individuals, it is not known if the quantity of calcification tracks the quantity of atherosclerosis over time in the same individuals. Further research is needed to better elucidate the relation of calcification to the pathogenesis of both atherosclerosis and plaque rupture.

Finally, histopathological studies provide the most accurateclues to a better understanding of human coronary artery disease. With better insight into disease pathophysiology, novel interventions could be introduced to improve care and future outcomes for patients undergoing coronary artery disease.

## Abbreviations

CAD: Coronary artery disease
CAC: Coronary artery calcium
SCD: Sudden coronary death
AMI: Acute myocardial infarction

## References

[1] Bairey NCB, Merz BD, Johnson BL, Sharaf WISE (2003). Hypoestrogenemia of hypothalamic origin and coronary artery disease in premenopausal women: a report from the NHLBI-sponsored WISE study. J Am Coll Cardiol.

[2] Chirinos JA, Segers P, Duprez DA, Brumback L, Bluemke DA, Zamani P, Kronmal R, Vaidya D (2015). Late systolic central hypertension as a predictor of incident heart failure: the Multi-ethnic Study of Atherosclerosis. J Am Heart Assoc.

[3] Bertomeu A, García-Vidal O, Farré X (2003). Preclinical coronary atherosclerosis in a population with low incidence of myocardial infarction: cross sectional autopsy study. British Med J.

The article "A histopathological analysis of the epidemiology of coronary atherosclerosis: an autopsy study" was retracted in 2016. Reasons: plagiarized text; compromised peer review; false authorship.

[4] Sharma K, Gulati M (2013). Coronary artery disease in women: a 2013 update. Glob Heart.

[5] Koopal C, Retterstøl K, Sjouke B, Hovingh GK, Ros E, de Graaf J, Dullaart RP (2015). Vascular risk factors, vascular disease, lipids and lipid targets in patients with familial dysbetalipoproteinemia: a European cross-sectional study. Atherosclerosis.

[6] Tintut Y, Patel J, Territo M (2002). Calcification of human vascular cells in vitro is correlated with high levels of matrix Gla protein and low levels of osteopontin expression. Circulation.

[7] Rodríguez-Saldaña J, Rodriguez-Flores M, Cantú-Brito C, Aguirre-Garcia J. A pathological study of the epidemiology of atherosclerosis in Mexico city. Cardiol Res Pract. 2014; doi:10.1155/2014/264205.10.1155/2014/264205PMC395563324719773

[8] Campbell LA, Rosenfeld ME. Infection and Atherosclerosis Development. Arch Med Res. 2015 May 2110.1016/j.arcmed.2015.05.006PMC452450626004263

[9] Rodrigues AN, Perez AJ, Carletti L, Bissoli NS, Abreu GR (2007). The association between cardiorespiratory fitness and cardiovascular risk in adolescents. J Pediatr (Rio J)..

[10] Knuiman MW, Folsom AR, Chambless LE, Liao D, Wu KK (2001). Association of hemostatic variables with MRI-detected cerebral abnormalities: the atherosclerosis risk in communities study. Neuroepidemiology.

[11] Jefferis BJ, Whincup PH, Lennon LT, Papacosta O, Goya WS (2014). Physical activity in older men: longitudinal associations with inflammatory and hemostatic biomarkers, N-terminal pro-brain natriuretic peptide, and onset of coronary heart disease and mortality. J Am Geriatr Soc.

[12] Wong TY, Klein R, Sharrett AR (2002). Retinal arteriolar narrowing and risk of coronary heart disease in men and women. The Atherosclerosis Risk in Communities Study. JAMA.

[13] Huber SA, Sakkinen P, David C (2001). T helper-cell phenotype regulates atherosclerosis in mice under conditions of mild hypercholesterolemia. Circulation.

[14] Gauss S, Klinghammer L, Steinhoff A, Raaz-Schrauder D, Marwan M, Achenbach S, Garlichs CD (2015). Association of systemic inflammation with epicardial fat and coronary artery calcification. Inflamm Res.

[15] Lakoski SG, Greenland P, Wong ND (2007). Coronary artery calcium scores and risk for cardiovascular events in women classified as “low risk” based on Framingham risk score: the Multi-Ethnic Study of Atherosclerosis (MESA). Arch Intern Med.

[16] de Oliveira Otto MC, Wu JH, Baylin A, Vaidya D, Rich SS, Tsai MY, Jacobs DR, Mozaffarian D (2013). Circulating and dietary omega-3 and omega-6 polyunsaturated fatty acids and incidence of CVD in the Multi-Ethnic Study of Atherosclerosis. J Am Heart Assoc.

The article "A histopathological analysis of the epidemiology of coronary atherosclerosis: an autopsy study" was retracted in 2016. Reasons: plagiarized text; compromised peer review; false authorship.

[17] Karakas M, Baumert J, Herder C, Rottbauer W, Meisinger C, Koenig W, Thorand B (2011). Soluble thrombomodulin in coronary heart disease: lack of an association in the MONICA/KORA case-cohort study. J Thromb Haemost.

[18] Mosca L, Benjamin EJ, Berra K, Bezanson JL, Dolor RJ, Lloyd-Jones DM, Newby LK (2011). Effectiveness-based guidelines for the prevention of cardiovascular disease in women–2011 update: a guideline from the American Heart Association. Circulation.

[19] Bielak LF, Yu P, Ryan KA, Rumberger JA, Sheedy PF, Turner ST, Post W, Shuldiner AR, Mitchell BD, Peyser PA (2008). Differences in prevalence and severity of coronary artery calcification between two non-Hispanic white populations with diverse lifestyles. Atherosclerosis.

[20] Newman AB, Naydeck BL, Whittle J (2002). Racial differences in coronary calcification in older adults. Arterioscl Thromb Vasc Biol.

[21] Budoff MJ (2003). Atherosclerosis imaging in calcified plaque: coronary artery risk assessment. Prog Cardiovasc Dis.

[22] Anaka A, Shimada K, Namba M (2008). Relationship between longitudinal morphology of ruptured plaques and TIMI flow grade in acute coronary syndrome: a three-dimensional intravascular ultrasound imaging study. Eur Heart J.

[23] Virmani R, Burke AP, Farb A, Gold HK, Finn AV, Kolodgie F (2007). Plaque rupture.Virmani R. The Vulnerable Atherosclerotic Plaque 2007.

[24] He ZX, Hedrick TD, Pratt CM (2000). Severity of coronary artery calcification by electron beam computed tomography predicts silent myocardial ischemia. Circulation.

[25] Mollet N, Maffei E, Martini C, Weustink A, van Mieghem C, Baks T, McFadden E, de Feyter P (2011). Coronary plaque burden in patients with stable and unstable coronary artery disease using multislice CT coronary angiography. Radiol Med.

[26] Bavelaar FJ, Beynen AC (2004). Atherosclerosis in parrots: a review. Vet Q.

[27] Brunkwall J, Mattsson E, Bergqvist D (1992). Diet-induced atherosclerosis in rabbits alters vascular prostacyclin release. Eicosanoids.

[28] Fricke C, Schmidt V, Cramer K (2009). Characterization of atherosclerosis by histochemical and immunohistochemical methods in African grey parrots (Psittacus erithacus) and Amazon parrots (Amazona spp.). Avian Dis.

[29] Centers for Disease Control and Prevention CDC (2005). Racial/ethnic and socioeconomic disparities in multiple risk factors for heart disease and stroke. MMWR Morb Mortal Wkly Rep.

[30] Galkina E, Ley K (2009). Immune and inflammatory mechanisms of atherosclerosis. Annu Rev Immunol.

[31] Hansson GK, Libby P (2006). The immune response in atherosclerosis: a double-edged sword. Nat Rev Immunol.

The article "A histopathological analysis of the epidemiology of coronary atherosclerosis: an autopsy study" was retracted in 2016. Reasons: plagiarized text; compromised peer review; false authorship.

[32] Kensey KR, Cho YI (2001). The Origin of Atherosclerosis: An Introduction to Hemodynamics.

[33] Greenland P, Alpert JS, Beller GA, Benjamin EJ, Budoff MJ, Fayad ZA, Foster E, Hlatky MA (2010). ACCF/AHA guideline for assessment of cardiovascular risk in asymptomatic adults: a report of the American College of Cardiology Foundation/American Heart Association Task Force on Practice Guidelines. J Am Coll Cardiol.

[34] Silverman S, Mader DR (2006). Diagnostic Imaging. Reptile Medicine and Surgery.

[35] Willecke F, Yuan C, Oka K, Chan L, Hu Y, Barnhart S, Bornfeldt KE, Goldberg IJ, Fisher EA (2015). Effects of High Fat Feeding and Diabetes on Regression of Atherosclerosis Induced by Low-Density Lipoprotein Receptor Gene Therapy in LDL Receptor-Deficient Mice. PLoS One.

[36] Smith SC, Smith EC, Taylor RL (2001). Susceptibility to spontaneous atherosclerosis in pigeons: an autosomal recessive trait.J. Heredity.

[37] Stetter MD, Mader DR (2006). Ultrasonography. Reptile Medicine and Surgery.

[38] Pearson TA, Blair SN, Daniels SR, Eckel RH, Fair JM, Fortmann SP (2002). AHA guidelines for primary prevention of cardiovascular disease and stroke: 2002 update: Consensus panel guide t comprehensive risk reduction for adult patients without coronary or other atherosclerotic vascular diseases. American Heart Association Science Advisory and Coordinating Committee. Circulation.

[39] Yusuf S, Reddy S, Ôunpuu S, Anand S (2001). Global Burden of Cardiovascular Diseases Part II: Variations in Cardiovascular Disease by Specific Ethnic Groups and Geographic Regions and Prevention Strategies. Circulation..

[40] Ford ES (2003). C-reactive protein concentration and cardiovascular disease risk factors in children: findings from the National Health and Nutrition Examination Survey 1999–2000. Circulation..

[41] Thomas AC, Knapman PA, Kirkler DA, Davies MJ (1988). Community study of the causes of ‘natural’ sudden death. Br Med J..

[42] Alioglu E, Turk UO, Engin C, Tengiz I, Tuzun N, Posacioglu H (2009). Left main coronary artery aneurysm in young patient with acute myocardial infarction. J Cardiovasc Med (Hagerstown).

[43] Hassantash SA, Bikdeli B, Kalantarian S, Sadeghian M, Afshar H (2008). Pathophysiology of aortocoronary saphenous vein bypass graft disease. Asian Cardiovasc Thorac Ann.

[44] Van der Wal AC, Becker AE, Elbers JRJ, Das PK (1992). An immunocytochemical analysis of rapidly progressive atherosclerosis in human vein grafts. Eur J Cardiothorac Surg.

[45] Leonard S. Lilly MD Pathophysiology of Heart Disease. A Collaborative Project of Medical Students and Faculty (Pathophysiology of heart disease (lilly)). Fifth Edition, North American Edition, ISBN-13: 978-1605477237

The article "A histopathological analysis of the epidemiology of coronary atherosclerosis: an autopsy study" was retracted in 2016. Reasons: plagiarized text; compromised peer review; false authorship.

[46] Packard RR, Lichtman AH, Libby P (2009). Innate and adaptive immunity in atherosclerosis. Semin Immunopathol.

[47] Cherian SM, Bobryshev YV, Inder SJ, Wang AY, Lord RS, Farnsworth AE (2000). Dendritic cells in aortocoronary saphenous vein bypass grafts. Heart Lung Circ.

[48] Thej MJ, Kalyani R, Kiran J (2012). Atherosclerosis in coronary artery and aorta in a semi-urban population by applying modified American Heart Association classification of atherosclerosis: An autopsy study. J Cardiovasc Dis Res.

[49] Yazdi SAT, Rezaei A, Azari JB, Hejazi A (2009). Prevalence of Atherosclerotic Plaques in Autopsy Cases with Noncardiac Death. Iranian J Pathol.

[50] Singh H, Oberoi SS, Gorea RK, Bal MS (2005). Atherosclerosis in coronaries in Malwa region of Punjab. JIAFM.

[51] Hassantash SA, Bikdeli B, Kalantarian S, Sadeghian M, Afshar H (2008). Pathophysiology of aortocoronary saphenous vein bypasses graft disease. Asian Cardiovasc Thorac Ann.

[52] Wong ND (2014). Epidemiological studies of CHD and the evolution of preventive cardiology. Nature reviews Cardiology.

[53] Rumberger JA, Brundage BH, Rader DJ, Kondos G (1999). Electron beam computed tomographic coronary calcium scanning: a review and guidelines for use in asymptomatic persons. Mayo Clin Proc..

[54] Deb S, Wijeysundera HC, Ko DT, Tsubota H, Hill S, Fremes SE (2013). Coronary artery bypass graft surgery vs percutaneous interventions in coronary revascularization: a systematic review. JAMA.

[55] Taylor AJ, Burke AP, O’Malley PG (2000). A comparison of the Framingham risk index, coronary artery calcification, and culprit plaque morphology in sudden cardiac death. Circulation.

[56] Assemat P, Siu KK, Armitage JA, Hokke SN, Dart A, Chin-Dusting J, Hourigan K (2014). Haemodynamical stress in mouse aortic arch with atherosclerotic plaques: preliminary study of plaque progression. Comput Struct Biotechnol J.

[57] Soraya H, Rameshrad M, Mokarizadeh A, Garjani A (2015). Metformin attenuates myocardial remodeling and neutrophil recruitment after myocardial infarction in rat. Bioimpacts.

[58] Mokarizadeh A, Hassanzadeh K, Abdi M, Soraya H, Faryabi MR, Mohammadi E, et. al. Trasnsdermal delivery of bovine milk vesicles in patients with multiple sclerosis: A novel strategy to induce MOG-specific tolerance. Med Hypotheses. 2015 Apr 2410.1016/j.mehy.2015.04.01925986518

[59] Mokarizadeh A, Delirezh N, Morshedi A, Mosayebi G, Farshid AA, Mardani K (2012). Microvesicles derived from mesenchymal stem cells: potent organelles for induction of tolerogenic signaling. Immunol Lett.

